The article "Mediating effect of self-esteem on the relationship between academic self-efficacy and depression symptoms among nursing students participating in blended learning" was retracted in 2025. Reasons: unreliable results or conclusions; concerns about the citations.

# Mediating effect of self-esteem on the relationship between academic self-efficacy and depression symptoms among nursing students participating in blended learning

**DOI:** 10.1016/j.heliyon.2023.e22526

**Published:** 2023-11-19

**Authors:** Bayu Fandhi Achmad, Akbar Satria Fitriawan, Dedi Kurniawan, Hsing-Mei Chen

**Affiliations:** a Department of Basic and Emergency Nursing, Faculty of Medicine, Public Health and Nursing, Universitas Gadjah Mada, Yogyakarta, Indonesia; b Department of Nursing, Faculty of Health Sciences, Universitas Respati Yogyakarta, Yogyakarta, Indonesia; c Department of Nursing, Kepanjen School of Health Sciences, Malang, East Java, Indonesia; d Department of Nursing, College of Medicine, National Cheng Kung University, Tainan, Taiwan

**Keywords:** Academic self-efficacy, Blended learning, Depression symptoms, Self-esteem

## Abstract

**Background:**

Blended learning, which comprises a combination of online and classroom-based activities, in nursing education can cause significant academic stress and depression symptoms among students. However, self-esteem may mediate the relationship between academic self-efficacy and depression symptoms. Studies of the relationship between academic self-efficacy, self-esteem, and depression symptoms among nursing students participating in blended learning are limited.

**Objectives:**

To examine the determinants of depression symptoms and the mediating effect of self-esteem on the relationship between academic self-efficacy and depression symptoms among nursing students who participate in blended learning.

**Design:**

Cross-sectional study using convenience sampling.

**Settings:**

Ten universities across five provinces and two major Indonesian islands.

**Participants:**

A total of 534 undergraduate nursing students with a mean age of 20.30 years (standard deviation, ±1.36 years).

**Methods:**

An online survey was conducted between April and August 2022 to collect data from 10 universities applying blended learning. The study instruments included the General Self-Efficacy Scale, Rosenberg Self-Esteem Scale, and a 9-item Patient Health Questionnaire. Data were analysed by hierarchical linear regression using PROCESS macro version 4.1.

**Results:**

Of the 534 participants, 213 (39.14 %) experienced moderate-to-severe depression symptoms. Two variables, online learning difficulties (β = 0.10; p = .012) and self-esteem (β = −0.40; p < .001), were significant determinants of depression symptoms. Self-esteem mediated the relationship between academic self-efficacy and depression symptoms.

**Conclusions:**

It is necessary to understand the online learning difficulties experienced by blended learning students and improve their self-esteem by maximising academic self-efficacy to prevent depression symptoms.

The article "Mediating effect of self-esteem on the relationship between academic self-efficacy and depression symptoms among nursing students participating in blended learning" was retracted in 2025. Reasons: unreliable results or conclusions; concerns about the citations.

## 1 Introduction

Blended learning is a deliberate combination of online and classroom-based activities that activate and support learning [1]. It has several positive effects, such as flexible learning, increased student engagement, and enhanced self-regulated learning [2,3]. However, it also comprises challenges and disadvantages for students, such as limited collaborative learning [4], lack of technological mastery [5], and low academic satisfaction [6]. During the coronavirus disease 2019 (COVID-19) pandemic, the majority of nursing education faculty began applying blended learning strategies to continue their education courses. Blended learning, however, has led to fewer opportunities for face-to-face learning and hands-on skills, thereby causing enormous academic stress [7] and depression symptoms [8] among students. Therefore, blended learning may require students to adjust their learning habits.

The prevalence of depression symptoms among nursing students during the COVID-19 pandemic was between 40 % and 50 % [9,10], which is higher than that reported before the COVID-19 pandemic (34 %) [11]. However, studies conducted both before and during the COVID-19 pandemic found similar factors associated with depression symptoms, including age [12], sex [13], financial problems [14], self-efficacy [15], academic grades [12], and satisfaction with grade point average (GPA) [15] among nursing students. These factors should be considered covariates or confounding factors when examining the significant determinants of depression symptoms, however, because the higher prevalence of depression symptoms during the pandemic may be related to other factors.

Depression symptoms have a considerable negative impact on the academic performance of nursing students [16]. Students with depression have difficulties with concentrating, problem-solving, and decision-making [17]. Consequently, they have a poor understanding of course materials, high absenteeism from classes, and lower academic performance, which may lead to the abandonment of studies [10]. However, depression symptoms can be prevented by increasing students’ self-esteem [18].

Self-esteem can be an individual's overall appraisal of oneself, personal beliefs, or perception of how one is appreciated in the social world [19]. Self-esteem plays a pivotal role in students' mental health because it may serve as a psychological buffer against depression [13]. Students with high self-esteem are more likely to have positive self-feelings, which help them manage unsatisfactory conditions [19], thereby preventing depression symptoms [20]. However, during the COVID-19 pandemic, students' self-esteem decreased because online learning created gaps between their social classes [15]. Students in low social classes may have insufficient equipment for online learning, which could make them feel embarrassed.

The article "Mediating effect of self-esteem on the relationship between academic self-efficacy and depression symptoms among nursing students participating in blended learning" was retracted in 2025. Reasons: unreliable results or conclusions; concerns about the citations.

Several studies have found that greater self-esteem is correlated with higher academic self-efficacy among students [[21], [22], [23]]. Those studies have shown that students who manage the adjustment process have higher academic self-efficacy and greater self-confidence and self-esteem regarding accomplishing their planned educational goals [21,22]. They also experience fewer depression symptoms [23]. However, the role of self-esteem in the relationship between academic self-efficacy and depression symptoms among nursing students remains unclear.

Although blended learning was a common and valuable alternative teaching strategy during the COVID-19 pandemic, it also caused stress for students. As mentioned, students with a low socioeconomic status may have insufficient computer equipment, access networks, or a room to work in, that can lead to lower academic self-efficacy [24] and undermine their self-esteem [25], further causing depression symptoms. However, studies investigating the relationship between academic self-efficacy, self-esteem, and depression symptoms among nursing students participating in blended learning are limited. Therefore, this study aimed to examine the determining factors of depression symptoms and the mediating effects of self-esteem on the relationship between academic self-efficacy and depression symptoms among nursing students participating in blended learning. We hypothesised that self-esteem would mediate the relationship between academic self-efficacy and depression symptoms.

## 2 Methods

### 2.1 Study design and setting

A quantitative cross-sectional design with an online questionnaire survey was used for this study. Participants were recruited from nationally accredited universities in Indonesia that offered blended learning courses for the first time during the COVID-19 pandemic.

### 2.2 Sample

The study employed a convenience sampling method. The inclusion criteria were undergraduate nursing students from the first to fourth academic years (the Bachelor of Nursing program in Indonesia is a 4-year program); participated in blended learning, especially in at least one of the three courses, including medical surgical nursing, pediatric nursing, or maternity nursing; and used a learning management system based on Moodle for communication, content distribution, and digital resources. The students taking academic leave were excluded. The minimum sample size was determined using G*Power software version 3.1.9.6 (Heinrich-Heine-Universität Düsseldorf, Düsseldorf, Germany) via a linear multiple regression analysis with the following assumptions: significance level p < .05; power = .80; Cohen's d effect size = 0.04 [26]; and nine predictor variables. A minimum sample of 400 participants was estimated.

The article "Mediating effect of self-esteem on the relationship between academic self-efficacy and depression symptoms among nursing students participating in blended learning" was retracted in 2025. Reasons: unreliable results or conclusions; concerns about the citations.

### 2.3 Instruments

The study instruments included demographic and academic performance data, the General Self-Efficacy Scale (GSE), the Rosenberg Self-Esteem Scale (RSES), and the nine-item Patient Health Questionnaire (PHQ-9). We have obtained permission to use the instruments before data collection. The demographic data included age and sex. Academic performance data included university type, academic grade, online learning difficulties (yes/no), financial problems during blended learning (yes/no), and satisfaction with GPA (yes/no).

Self-efficacy was measured using the GSE developed by Jerusalem and Schwarzer (1979) [27]. The GSE consists of 10 items rated using a 4-point Likert scale as follows: strongly disagree, 1; disagree, 2; agree, 3; and strongly agree, 4. The total score ranges from 10 to 40. Higher scores indicate higher self-efficacy [28]. This study used the Indonesian version of the GSE translated and validated by Putra et al. [29]. Cronbach's α for internal consistency reliability was 0.87 for the original version of the GSE [27] and 0.85 for this study.

Self-esteem was assessed using the RSES developed by Rosenberg in 1965 [30]. The RSES consists of 10 items (five positive statements and five negative statements) with four possible answers rated using a Likert scale. For the positive statements (items 1, 3, 4, 7, and 10), the answers were rated as follows: strongly disagree, 1; disagree, 2; agree, 3; and strongly agree, 4. The answers for the negative statements (items 2, 5, 6, 8, and 9) were reverse-coded [31]. The total score ranges from 10 to 40 and is categorised into three levels: low self-esteem, 10–25; moderate self-esteem, 26–29; and high self-esteem, 30–40 [32]. This study used the Indonesian version of the RSES translated and validated by Maroqi [33]. Cronbach's α was 0.73 for the original version of the RSES [30] and 0.82 for this study.

The PHQ-9 was used to assess depression symptoms [34]. The PHQ-9 consists of nine items with four answer choices with scores ranging from 0 (never) to 3 (almost every day). The total PHQ-9 score ranges from 0 to 27 [35]. This study used the Indonesian version of the PHQ-9 translated and validated by Dian et al. [36]. Cronbach's α was 0.85 for the original version of the PHQ-9 [34] and 0.89 for this study.

The article "Mediating effect of self-esteem on the relationship between academic self-efficacy and depression symptoms among nursing students participating in blended learning" was retracted in 2025. Reasons: unreliable results or conclusions; concerns about the citations.

### 2.4 Ethical consideration

Ethical clearance was obtained from the Health Research Ethics Committee, Universitas Respati Yogyakarta, Indonesia (ethical number: 239.3/FIKES/PL/XII/2021 on 29 December 2021). We used the Declaration of Helsinki on Biomedical Research Involving Human Subjects as a guideline for this study. Informed consent was obtained from each participant before data collection. The confidentiality of all the information obtained from the participants was assured throughout the study.

### 2.5 Data collection procedure

Data were collected from April to August 2022. The researchers searched all the nationally accredited universities in Indonesia that offered blended learning during the COVID-19 pandemic by checking the curricula on university websites. An email was sent to potential universities to confirm their use of blended learning. A research approval letter was obtained from universities that met the eligibility criteria. Next, the universities were asked to help screen and send the researchers’ study information to the undergraduate nursing students. The researchers emailed the students to confirm their eligibility and obtained informed consent if they met the inclusion criteria. Finally, students received a link to the online questionnaires using Google Forms. A “required” command for each item was created to prevent students from missing an answer (a “not applicable” response was used for those who did not have an answer for certain items); therefore, there were no missing data to be replaced (Fig. 1).

**Fig. 1:** Flowchart of study participants.

### 2.6 Statistical analysis

IBM SPSS version 21 (IBM Corp., Armonk, NY, USA) was used for the data analysis. Descriptive statistics of categorical variables are presented as frequencies and percentages. Numerical variables were presented as means and standard deviations. In the present study, the data were not normally distributed. Based on the large sample size (n = 534), parametric analyses were performed based on the central limit theorem [37]. An independent *t*-test was performed to investigate the association between depression symptoms and factors in two categories, whereas a one-way analysis of variance was performed for variables in more than two categories. Pearson's correlation was used to analyse depression and continuous independent variables. The results were cross-validated using a non-parametric analysis.

A multiple linear regression analysis and hierarchical method were used to identify major factors associated with depression symptoms. Variables that showed an association (p < .25) with depression symptoms in the bivariate analysis were included in the regression model. Subsequently, a four-step hierarchical linear regression involving eight variables was performed. We adapted Bandura's self-efficacy theory to include the variables in the model [38]. The first step of the analysis involved demographic factors, including age and sex (model 1). Next, academic performance factors, including three dummy variables for grades, financial problems, online learning difficulties, and satisfaction with GPA, were added during the second step (model 2). Academic self-efficacy was included during the third step (model 3). Finally, self-esteem was included during the fourth step (model 4). Additionally, we used PROCESS macro version 4.1 (Canadian Centre for Research Analysis and Methods, Calgary, Alberta, Canada) to analyse the role of self-esteem in the relationship between academic self-efficacy and depression symptoms. A 95 % bias-corrected confidence interval (CI) was created using bootstrapping with 5000 resamples, and model 4 was applied to examine the serial mediating effect.

The article "Mediating effect of self-esteem on the relationship between academic self-efficacy and depression symptoms among nursing students participating in blended learning" was retracted in 2025. Reasons: unreliable results or conclusions; concerns about the citations.

## 3 Results

Ten universities responded to our email and confirmed the implementation of blended learning in their curricula. A total of 534 of 3687 undergraduate nursing students completed the study questionnaires. The average age of participants was 20.30 years (standard deviation, ±1.36 years; range, 18–24 years). Most participants reported financial problems, especially regarding online learning, during the COVID-19 pandemic (n = 423; 79.21 %) and had difficulties attending online learning courses (n = 416; 77.90 %). The participants’ average academic self-efficacy was 30.64 (standard deviation, 4.40). More than half of the participants had high self-esteem (n = 296; 55.43 %). Additionally, most of the participants reported mild depression symptoms (n = 213; 39.89 %). Detailed information regarding the sociodemographic characteristics of participants and major variables is provided in Fig. 2 and Table 1.

**Fig. 2:** Participants' characteristics (N = 534) Notes. OL: online learning; GPA: grade point average.

**Table 1:** Distribution of major variables of depression symptoms (N = 534).

Characteristics	*M*	SD
Age (years)	20.30	1.36
Academic self-efficacy	30.64	4.40
Self-esteem	30.14	4.05
Depression status	8.87	5.37

Notes. *M*: mean; SD: standard deviation.

As shown in Table 2, Table 3, bivariate statistical analyses revealed that six variables, sex (t = −2.42; p = .016), financial problems (t = 2.67; p = .008), online learning difficulties (t = 2.83; p = .005), satisfaction with GPA (t = 2.36; p = .019), self-esteem (r = −0.46; p < .001), and academic self-efficacy (r = −0.27; p < .001), were significantly associated with depression symptoms. Considering the multicollinearity effects among variables, eight variables that showed an association with depression symptoms with a significance level of p < .25 [39] in the bivariate analysis were included in the four-step regression model (Table 4). During step 1, demographic variables including age and sex were included in the model analysis (model 1). The results showed that sex was an important factor influencing depression symptoms (β = 0.09; p = .039). The R^2^ value of the model was 0.014. During step 2, academic performance factors, including grades, financial problems, online learning difficulties, and satisfaction with GPA, were analysed (model 2). The results showed that financial problems (β = 0.09; p = .040) and online learning difficulties (β = 0.10; p = .032) were significant factors, with a significant increase in the R^2^ value compared to that of model 1 (R^2^ = 0.05; ΔR^2^ = 0.03; p = .001). During step 3, academic self-efficacy was added (model 3). The findings showed that online learning difficulties (β = 0.10; p = .016) and academic self-efficacy (β = −0.27; p < .001) were two significant factors associated with depression symptoms, with a significant increase in the R^2^ value compared to that of model 2 (R^2^ = 0.12; ΔR^2^ = 0.07; p < .001). Finally, self-esteem was included in the regression model (model 4). The results showed that online learning difficulties (β = 0.10; p = .012) and self-esteem (β = −0.40; p < .001) were two determinant factors, with a significant increase in the R^2^ value compared to that of model 3 (R^2^ = 0.24; ΔR^2^ = 0.12; p < .001).

The article "Mediating effect of self-esteem on the relationship between academic self-efficacy and depression symptoms among nursing students participating in blended learning" was retracted in 2025. Reasons: unreliable results or conclusions; concerns about the citations.

**Table 2:** Bivariate analysis of categorical variables associated with depression symptoms (N = 534).

Characteristics	Depression symptoms		
	*M* ± SD	*t*/*F*	p
Sex		−2.42	.016*
Male	7.51 ± 5.34		
Female	9.10 ± 5.35		
Type of university		−.19	.853
Private	8.86 ± 5.36		
Public	9.00 ± 5.55		
Grades		1.83	.141
First-year	9.55 ± 5.32		
Second year	8.33 ± 5.14		
Third year	8.68 ± 5.69		
Fourth-year	8.35 ± 5.29		
Financial problems		2.67	.008**
Yes	9.19 ± 5.45		
No	7.67 ± 4.93		
Online learning difficulties		2.83	.005**
Yes	9.22 ± 5.46		
No	7.64 ± 4.89		
Satisfaction with GPA		2.36	.019*
No	9.28 ± 5.40		
Yes	8.14 ± 5.26		

Notes. *p < .05; **p < .01; ***p < .001; Independent t-tests for two-categorical variables; One-way analysis of variance for three- and more categorical variables; GPA: grade point average.

**Table 3:** Relationship between continuous variables and depression symptoms.

	1	2	3	4
Age	1			
Self-esteem	.07	1		
ASE	−.02	.49***	1	
Depression	−.08	−.46***	−.27***	1

*p < .05; **p < .01; ***p < .001; ASE: academic self-efficacy.

Note: p-value for the relationship between age and depression is p = .066.

The article "Mediating effect of self-esteem on the relationship between academic self-efficacy and depression symptoms among nursing students participating in blended learning" was retracted in 2025. Reasons: unreliable results or conclusions; concerns about the citations.

**Table 4:** Hierarchical Regression of Predictors variables on depression symptoms.

Variable	Step 1		Step 2		Step 3		Step 4	
	β	t	β	t	β	t	β	t
Age	−.06	−1.34	−.05	−.74	−.02	−.34	−.01	−.22
Sex	.09	2.07*	.08	1.75	.07	1.70	.05	1.25
Second year^1^			−.09	−1.69	−.09	−1.83	−.06	−1.42
Third year^1^			−.04	−.60	−.08	−1.31	−.06	−1.08
Fourth year^1^			−.04	−.64	−.08	−1.24	−.05	−.87
Financial problems			.09	2.06*	.07	1.74	.06	1.43
Online learning difficulties			.10	2.15*	.10	2.42*	.10	2.51*
GPA satisfaction			−.07	−1.52	−.07	−1.59	−.05	−1.37
ASE					−.27	−6.52***	−.07	−1.66
Self-esteem							−.40	−9.17***
F		3.84		3.32		7.91		16.7
*R*^*2*^		.014*		.048		.120		.242
*R*^*2*^ change		.014		.034**		.072***		.122***
Adjusted *R*^*2*^		.011		.034		.104		.227

Notes. *p < .05; **p < .01; ***p < .001; ^1^Reference group: first year; GPA: grade point average.

A mediation analysis showed that academic self-efficacy was significantly associated with self-esteem (β = 0.45; p < .001) and depression symptoms (β = −0.33; p < .001). When self-esteem was included in the PROCESS macro as a mediator variable, the relationship between self-esteem and depression symptoms was significant (β = −.57; p < .001), but the relationship between academic self-efficacy and depression symptoms became non-significant (β = −.07; p = .098) (Fig. 3). The indirect effect of academic self-efficacy on depression symptoms was −0.25, and the bootstrap CI did not reach zero (95 % CI = −0.36 to −0.17). The results indicated a fully mediating effect of self-esteem on the relationship between academic self-efficacy and depression symptoms.

**Fig. 3:** Mediating effect of self-esteem on the relationship between academic self-efficacy and depression symptoms *p < .05; **p < .01; ***p < .001.

## 4 Discussion

This study showed that sex, financial problems, online learning difficulties, satisfaction with GPA, academic self-efficacy, and self-esteem were significantly associated with depression symptoms among students participating in blended learning. However, only online learning difficulties and self-esteem were found to be determinants. Similarly, self-esteem mediates the relationship between academic self-efficacy and depression symptoms.

Four of 10 nursing students participating in blended learning reported moderate-to-severe depression symptoms (Table 1). This number was lower than that reported by Kwak et al. [10] among nursing students during the COVID-19 pandemic, but it was higher than that reported before the COVID-19 pandemic [11]. However, the prevalence of depression symptoms among blended learning students is still higher than that among online learning students [14,40,41]. Villani et al. [42] argued that nursing students may develop depression symptoms because of the fear of returning to the university and COVID-19 infection after the confinement period. Furthermore, the demand to adapt to changing learning methods (online and offline) of each course is psychologically overwhelming for students, resulting in a loss of motivation and interest in learning [43], which can affect their learning engagement and academic achievement [7].

The article "Mediating effect of self-esteem on the relationship between academic self-efficacy and depression symptoms among nursing students participating in blended learning" was retracted in 2025. Reasons: unreliable results or conclusions; concerns about the citations.

Females were predominant in our study, where the results also showed higher depression symptoms than males. The findings are consistent with Johnson and Taliaferro [44], which stated that female students had 1.32 greater odds of experiencing symptoms of depression compared to males. The symptoms include depressed mood, anhedonia, sleep disturbances, guilt, fatigue, difficulty concentrating, changes in appetite, agitation, and suicidal thoughts. The difference in depression rates between males and females may indicate that females may have more difficulties to adjust to the stressful factors in university life [45].

Self-esteem was a significant determinant of depression symptoms in this study sample. A previous study supported the notion that self-esteem can influence the depression symptoms of students because it may serve as a psychological buffer against the development of depression disorder and hostility [13]. Similarly, another study revealed that psychopathological factors such as low self-esteem and hopelessness have an empirical relationship with depression symptoms [20]. Additionally, low self-esteem can predispose students to so-called vulnerability to depression, whereby they tend to create harsh self-criticisms and interpret specific mistakes as a reflection of their total failure [46].

Difficulty learning online was another determinant of depression symptoms among nursing students during the COVID-19 pandemic. Indonesian students are relatively new to blended learning. As a result, students were not only facing the COVID-19 pandemic but also facing the need to adjust to diverse learning methods. Mtebe and Raphael [47] reported that difficulties with information and communication technology skills are the most significant issues for students. Similarly, financial problems may impede their access to the technology needed to continue their online learning. Studies have emphasized the issue that students with barriers to obtaining electronic devices and a stable Internet connection for blended learning cause difficulty accessing information during online learning [14,48]. Therefore, a mastery of information and communication technology and adequate financial support are essential for participating in blended learning.

The article "Mediating effect of self-esteem on the relationship between academic self-efficacy and depression symptoms among nursing students participating in blended learning" was retracted in 2025. Reasons: unreliable results or conclusions; concerns about the citations.

During this study, academic self-efficacy was inversely correlated with depression symptoms, but it was not a determinant. Similarly, Esteban et al. [15] found that students with low academic self-efficacy were more likely to experience depression because they attributed their failure to their low academic ability. In contrast, students with high academic self-efficacy tend to see failure as an opportunity to increase their attempts to obtain better results. As mentioned, high academic self-efficacy was a protective factor against depression symptoms among nursing students [15]. Furthermore, low academic self-efficacy can cause students to fear completing their tasks, avoid tasks, postpone tasks, and quit, whereas high academic self-efficacy motivates them to persevere and face challenging situations, thereby preventing academic burnout and depression [49].

The study findings support the idea that self-esteem plays a mediating role in the relationship between academic self-efficacy and depression symptoms among nursing students participating in blended learning. These results imply that increasing students’ self-esteem can increase their academic self-efficacy, ultimately resulting in decreased depression symptoms. This finding is consistent with those of previous studies that reported that self-esteem is a protective mechanism against depression [19,50].

The substantial effects of academic self-efficacy on self-esteem may be attributable to increased academic performance and achievement, which can help students avoid negative judgments and critical thoughts, thus further enhancing their self-esteem [51]. Enhanced self-esteem acts as a buffer against depression symptoms among students. Individuals with higher academic self-efficacy are highly aware of positive academic emotions and use them as coping mechanisms for low self-esteem and depression symptoms [50]. Therefore, it is reasonable to infer that self-esteem mediates the relationship between academic self-efficacy and depression symptoms.

### 4.1 Study limitations

Although the findings of this study contribute significantly to our understanding of the relationship between academic self-efficacy, self-esteem, and depression symptoms among blended-learning students, some limitations should be considered. First, this study used self-report questionnaires as outcome measures, which might have increased the risk of social desirability bias. Future studies with mixed-method designs are required to explore students’ responses and provide supplementary information. Second, this study used a cross-sectional research design; therefore, a demonstration of the cause-and-effect relationship between the variables was not possible. Longitudinal studies may help provide a better understanding of the mediation model using these variables. Third, a convenience sampling method was adopted, which may have limited the generalizability of the findings. However, we believe that our large student sample, which included 10 universities across five provinces and two major islands, is representative of the academic problems experienced by nursing students in Indonesia. Further studies using stratified random sampling methods and involving multinational participants are required to increase the generalizability of the findings. Fourth, females were predominant in our study, which might affect the results of this study. The imbalance may be because there are more female nursing students than male students.

The article "Mediating effect of self-esteem on the relationship between academic self-efficacy and depression symptoms among nursing students participating in blended learning" was retracted in 2025. Reasons: unreliable results or conclusions; concerns about the citations.

## 5 Conclusions

A high prevalence of depression symptoms was observed among Indonesian nursing students during the COVID-19 pandemic. The study findings suggest the need to understand students’ online learning difficulties when participating in blended learning, particularly those of students with a low socioeconomic status. Helping students to become academically prepared by providing them with adequate equipment and a stable Internet connection for online learning without reducing their self-esteem is essential to preventing depression symptoms and maximising academic self-efficacy.

Course coordinators should help students overcome problems associated with online learning by providing appropriate feedback through live chats, emails, or phone calls. An online learning environment that allows all students to be actively involved, cultivates self-confidence, and provides respect for all students is required. Additionally, the university should provide learning centres equipped with computers with fast Internet connections for students who cannot afford online learning devices. Furthermore, teachers should record class sessions to ensure that course materials can be accessed later by students who experience unstable Internet connections. These methods can help students overcome online learning difficulties, improve self-efficacy, and sustain self-esteem, ultimately minimising the risk of depression symptoms.

## Data availability statement

Data will be made available on request.

## Funding

Indonesia Endowment Funds for Education (10.13039/501100014538LPDP) and Center for Higher Education Funding (BPPT) (202101120133).

## Additional information

No additional information is available for this paper.

## CRediT authorship contribution statement

**Bayu Fandhi Achmad:** Conceptualization, Data curation, Methodology, Project administration, Software, Writing – original draft, Writing – review & editing. **Akbar Satria Fitriawan:** Conceptualization, Data curation, Methodology, Project administration. **Dedi Kurniawan:** Data curation, Project administration, Software. **Hsing-Mei Chen:** Conceptualization, Formal analysis, Methodology, Supervision, Validation, Visualization, Writing – review & editing.

The article "Mediating effect of self-esteem on the relationship between academic self-efficacy and depression symptoms among nursing students participating in blended learning" was retracted in 2025. Reasons: unreliable results or conclusions; concerns about the citations.

## Declaration of competing interest

The authors declare that they have no known competing financial interests or personal relationships that could have appeared to influence the work reported in this paper.
